# Circular RNA KIF4A Promotes Liver Metastasis of Breast Cancer by Reprogramming Glucose Metabolism

**DOI:** 10.1155/2022/8035083

**Published:** 2022-08-23

**Authors:** Jun Huang, Xinpei Deng, Xuedong Chen, Zaoshang Chang, Quzhe Lu, Anliu Tang, Peng Liu

**Affiliations:** ^1^College of Basic Medicine, Shaoyang University, Shaoyang, China; ^2^Sun Yat-sen University Cancer Center, State Key Laboratory of Oncology in South China, Collaborative Innovation Center for Cancer Medicine, Guangzhou, China; ^3^Department of Gastroenterology, The Third Xiangya Hospital of Central South University, Changsha, China

## Abstract

**Background:**

Circular RNAs (circRNAs) regulate complex functional processes and play crucial roles in cancer development and progression. It was reported that circKIF4 regulates the progression of triple-negative breast cancer (TNBC). This study evaluates the role of circKIF4 in breast cancer distant metastasis and metabolic reprogramming.

**Methods:**

RT-qPCR was performed to verify the expression of circKIF4A in breast cancer, liver metastatic tissues, and cell lines. The function of circKIF4A in metastasis was evaluated both in vitro and in vivo through a series of experiments, including cell migration and glucose intake experiments. Additionally, we conducted molecular experiments to clarify the regulatory role of circKIF4A. We then conducted a Luciferase reporter assay and an RNA immunoprecipitation assay to identify the molecular interactions between circKIF4A and miRNA.

**Results:**

circKIF4A was overexpressed in breast cancer cell lines and tissues, inhibiting its expression and suppressing breast cancer growth and metastasis. Interestingly, we observed that circKIF4A reprogrammed the glucose metabolism of breast cancer, and silencing circKIF4A greatly affected glucose uptake and lactate production in breast cancer cells. miR-335 can be sponged by circKIF4A, which affected the expression of ALDOA/OCT4 protein and regulated HK2/PKM2 expression.

**Conclusions:**

This study demonstrated that the circKIF4A-miR-335-OCT4/ALDOA-HK2/PKM2 axis is critical to breast cancer metabolic reprogramming, indicating that this axis could be a novel therapeutic target for the treatment of liver metastasis of breast cancer.

## 1. Introduction

As the leading cause of cancer-related mortality among women, breast cancer (BC) is the most common malignancy affecting women worldwide [1]. A recent update on cancer statistics reveals that the overall survival rate for primary BC is approaching 99%. Unfortunately, distant metastases develop in approximately one-third of BC patients, decreasing their five-year survival rate to 28% for patients with distant metastases [2]. Liver, lung, brain, and bone are the most common sites for BC metastasis. As the third most common site of BC metastasis, liver metastasis is developed in half of BC patients with metastases, and 5% to 12% of BC patients develop liver metastases as their main organ of recurrence [3]. Patients with liver metastasis typically live between 4 and 8 months if they do not receive proper treatment [4]. For most patients with distant lymph node or liver metastasis, they have limited treatment options that are mostly systemic hormones or chemotherapy, which can only prolong their survival period to about 18–24 months, with a great burden of tumor cells and deterioration of liver function [5–7]. Currently, the mechanism of this life-threatening problem remains known. In this study, we aim to identify mechanisms and targets that could guide precise antimetastatic therapy for breast cancer.

Noncoding RNAs have vital regulating roles in cancer development and progression. Circular RNA (circRNA) is a type of intracellular noncoding RNA [8]. circRNAs are abundant in human cells without the structure of a 3′-tail or a 5′-head and are capable of modulating or affecting gene expression via a variety of mechanisms, including modulating transcription, regulating splicing, platforms for proteins, and sponges for miRNAs, and outcompeting linear mRNAs for protein binding [9, 10]. Since the advent of circRNA sequencing technology, especially high-throughput microarray sequencing, a growing number of circRNAs have been identified and shown to modulate various types of cancers [11–13]. CDR1AS/CIRS-7 is well known to block miRNA miR-7, facilitating tumor proliferation, immune evasion, metastasis, and resistance to chemo in diverse cancers [14–18]. In both glioma and breast cancer, circular RNA FBXW7 was found to inhibit the proliferation and migration of cells by encoding a 21 kDa/185aa peptide [19, 20]. circGNB1 upregulates IGF1R by spiking miR-141-5p and facilitating TNBC progression [21]. Additionally, circular RNA was found to be involved in regulating glucose metabolism. By sponging miR-516b, the silence of circRAD18 could decrease PDK1 expression, participate in the metabolic reprogramming of glucose in papillary thyroid cancer, and inhibit the cell glucose uptake and lactate production [22]. Breast cancer cells were also found to respond to CircRAD18 when they are blocked by miR-208a [23]. Using circular RNA microarrays, Hailin Tang et al. detected the differential circRNA expression in TNBC at the molecular level and discovered that circKIF4A in TNBC tissue may serve as a potential prognostic biomarker and a therapeutic target [24]. However, the mechanism of circKIF4A in liver metastatic involvement of breast cancer remains unclear.

In this study, we found that circKIF4A was differentially expressed in breast cancer and liver metastatic tissues and cells and involved in the promotion of liver metastasis and glucose production. Furthermore, molecular studies revealed that the circKIF4A-miR-335-OCT4/ALDOA-HK2/PKM2 axis participates in the metabolic reprogramming and progression of breast cancer.

## 2. Materials and Methods

### 2.1. Cell Culture

Normal breast epithelial cell line 184A1 and breast cancer cell lines MCF-7, BT-474, and HCC1806 were obtained from ATCC. Cells were cultured and passaged in a humidified incubator (Thermo Fisher Scientific, MA, USA) at 37°C with 5% CO_2_ for less than 6 months. All the cell lines were verified to be free of mycoplasma infection with DNA fingerprinting.

### 2.2. Patients and Samples

The primary breast cancer and liver metastases samples were collected from patients at the Sun Yat-Sen University Cancer Center (SYSUCC) in Guangzhou, China. Upon collection, all samples were immediately submerged in RNA later solution. The whole process of sample collection was approved by the institutional review committee. The samples were collected from patients with informed consent. After collection, the samples were stored at −4°C overnight, and then the RNA later was discarded and samples stored at −80°C until used.

### 2.3. RT-qPCR Analysis

All qRT-PCR analyses were performed with an SYBR Green qPCR Kit (Takara, Japan). The primers for circKIF4A were F: 5′- GAGGTACCCTGCCTGGATCT -3′ and R: 5′-TGGAATCTCTGTAGGGCACA-3′. The primers for KIF4A were F: 5′- AGCTTCTTTAATCCCGTCTGTG-3′ and R: 5′-GGCCAGAGCCCGTTTCTTT -3′. The primers for GAPDH were F: 5′-GGAGCGAGATCCCTCCAAAAT -3′ and R: 5′- GGCTGTTGTCATACTTCTCATGG -3′. The primers for 18 S were F: 5′- TTAATTCCGATAACGAACGAGA-3′ and R: 5′-CGCTGAGCCAGTCAGTGTAG -3′. The qRT-PCR plate was employed from NEST NO.402301.

### 2.4. RNase R Digestion Assay

Briefly, an extract of three micrograms of RNA from breast cancer cells was treated with RNase R (2 U/*μ*g) or distil water for 30 minutes at 37°C. The remaining RNA solution was used for qRT-PCR analysis.

### 2.5. Actinomycin D Digestion Assay

We digested the MCF-7, BT474, and HCC1806 breast cell lines with 5 *μ*g/ml actinomycin *D* (Sigma) at 0-hour, 8-hour, 16-hour, and 24-hour time points. A qRT-PCR analysis was then conducted on circKIF4A and linear host gene KIF4A mRNA.

### 2.6. Western Blot Analysis

Briefly, the total proteins were extracted from BC cells using RIPA lysis buffer, separated by SDS-PAGE, and subsequently transferred to PVDF membranes. After being blocked with 5% skim milk at room temperature for 1 h, the membrane was incubated with the primary antibody at 4°C overnight and then a secondary antibody was used at room temperature for 1 hour and detected by chemiluminescence. The primary antibodies 1: 1000 anti-ALDOA (CST) and 1 : 3000 anti-GAPDH-actin (Abcam) were used in this study.

### 2.7. Transwell Assay

5 × 10^4^ cells were digested and resuspended. Cells from each group were added to the superior chambers (without FBS) and lower cross-pore compartment (containing 20% FBS). After 22 hours, we imaged and counted all migrated BC cells after they were fixed with methanol and stained with crystal violet (2.5%).

### 2.8. Assessment of Glucose Intake and Lactate Production

For measuring the consumption of glucose and production of lactate, we used the Amplex Red Glucose/Glucose Oxidase Assay Kit (Invitrogen, USA). In order to normalize the data, the amounts of total cellular protein were taken.

### 2.9. Luciferase Reporter Assay

3 × 10^3^ BC cells were seeded into 96-well plates. The predicted miR-335 binding sites of circKIF4A and the 3′-UTR of ALDOA mRNA were manually mutated. Then, reporting plasmids (circKIF4A-wt/mut or 3′-UTR of ALDOA-wt/mut) and mimics of certain miRNA were cotransfected using a Promega luciferase kit for 48 hours.

### 2.10. RNA Immunoprecipitation (RIP)

In this assay, the AGO2 antibody (CST, USA) was used. We detected the relative expression levels of circKIF4A, miR-335, and ALDOA mRNA after RNA purification. RIP assays were conducted after 72 hours of incubation of breast cancer cells transfected with MS2-Rluc.

### 2.11. Animal Experiments

All animal procedures and care were conducted in accordance with institutional guidelines with the approval of SYSUCC's Institute Research Ethics Committee. The liver metastasis experiments were performed using 1 × 10^6^ BC cells stably overexpressing circKIF4A that were injected into the spleens of female BALB/*c* mice; control cells were injected into other mice. We euthanized the mice after 60 days and removed the livers for pathological assessment. Metastatic nodules in the liver were counted via visual examination and microscopy of hematoxylin and eosin (HE)-stained sections.

### 2.12. Statistical Analysis

All data analyses were performed with SPSS 24.0 software (IBM, SPSS, USA) and GraphPad Prism 9 (GraphPad Software Inc., USA). To compare expression between two matched groups, a paired Student's *t*-test was performed. Quantitative data are presented as mean ± standard deviation (SD) and *P* < 0.05 were considered as statistically significant.

## 3. Results

### 3.1. circKIF4A Is Overexpressed in Breast Cancer and Liver Metastasis with Circular RNA Structure

Based on the RT-qPCR analysis of noncancer, primary cancer, and liver metastasis tissues, it was found that circKIF4A was upregulated in primary cancer and liver metastasis samples (Figure 1(a)). Furthermore, circKIF4A was overexpressed in three breast cancer cell lines compared to 184A1 cells (Figure 1(b)). We examined the characteristics of circKIF4A with its degradation by RNase R resistant assays and actinomycin D digestion assays and found that circKIF4A was resistant to RNase R, while RNase R degraded the linear form of KIF4A mRNA (Figure 1(c)). Consistently, circKIF4A showed greater stability of circular structure in the three different breast carcinoma cell lines than linear KIF4A mRNA (Figure 1(d)).

### 3.2. Silence of circKIF4A Suppresses Glucose Metabolism and Prevents Breast Cancer Cells from Metastasis

After being transfected with siRNA, the silence of circKIF4A significantly inhibited glucose uptake and lactate production in breast cancer cells (Figures 2(a) and 2(b)). To determine whether circKIF4A is involved in breast cancer metastases, we performed migration and invasion assays, which showed that silencing circKIF4A reduced the migration of MCF-7, BT474, and HCC1806 cells in transwell assays (Figure 2(c)).

### 3.3. circKIF4A Is a Sponge for miR-335 in Breast Cancer

We performed qPCR analysis to determine the subcellular location of circKIF4A by isolating its cytoplasmic and nuclear components. The results indicated that circKIF4A was predominantly accumulated in the cytoplasm, where miRNA is generally found, suggesting that circKIF4A might interact with miRNA (Figure 3(a)). According to our predictions, miR-335 has the potential to bind to the binding elements of circKIF4A (Figure 3(b)). Moreover, dual luciferase reporter assays demonstrated that circKIF4A can interact with miR-335 (Figure 3(c)). To confirm this interaction, we performed MS2-related RNA immunoprecipitation assays on circKIF4A and miR-335, and the results revealed that miR-335 was remarkably elevated in the MS2-circKIF4A-wt group (Figure 3(d)). Transfecting cells with si-circ-KIF4A increased the expression of miR-335 as measured by RT-qPCR analysis (Figure 3(e)).

### 3.4. circKIF4A Regulates Breast Cancer Metabolism Reprogramming

Compared to 184A1 cells, miR-335 was downregulated in three BC cell lines (Figure 4(a)). RT-qPCR analysis revealed that miR-335 was downregulated in primary cancer and liver metastasis (Figure 4(b)). After transfected with miR-335 mimics, the glucose uptake and lactate production were reduced, indicating that miR-335 is involved in the glucose metabolism reprogramming (Figure 4(c)). Utilizing TargetScan, the miR-335 targets were predicted and its downstream effects were screened. ALDOA and POU5F1 (also called OCT4) were the top two molecules identified (Figure 4(d)). Both ALDOA and OCT4 are metabolic proteins associated with glucose intake [25, 26] and are crucial for cancer progression [27, 28]. It has been suggested that ALDOA and OCT4 regulate metabolism-related proteins, such as HK2 and PKM2 [29, 30]. The transfection of miR-335 mimics reduced the mRNA expression of ALDOA/HK2 and OCT4/PKM2 significantly (Figure 4(e)). Furthermore, mimicking miR-335 resulted in a reduction of ALDOA/HK2 and OCT4/PKM2 protein expression (Figure 4(f)).

To further evaluate how circKIF4A functions in liver metastasis, we injected BC cells stably overexpressing circKIF4A and the corresponding control cells into the inferior hemispleen to drive liver metastasis. A striking difference between the circKIF4A overexpression group and the control group was noted in the number of liver metastatic nodules (Figures 5(a)–5(c)). Furthermore, introduction of the circKIF4A mimics could increase glucose uptake and lactate production, which could be reversed by supplementation with miR-335.

## 4. Discussion

Worldwide, most of the deaths associated with BC occur from metastases, which account for over 90% of BC death cases [31]. The discovery of circRNAs, a large class of noncoding RNA in the past decade, has rapidly become a hot topic in research for the pathogenesis of cancers [32, 33]. Following the establishment of several famous circRNA databases in the past few years, a growing number of circRNAs have been identified and well studied as part of cancer research [33–35]. CDR1as/ciRS-7, the most well-known circRNA, was proved to sponge miR-7 and regulate proliferation, metastasis, and microenvironment of multiple cancers [14–18]. The tumor growth and metastasis of TNBC and glioma are inhibited by circFBXW7, which encodes protein FBXW7-185aa and blocks miR-197-3p [19, 20]. CircRNAs were found as tumor-promoting modules by promoting proliferation and reducing apoptosis in TNBC [21, 36]. Despite these findings, studies on the role of circRNAs in distant metastasis have been rare. In one research, CircANKS1B was found to be upregulated in TNBC and promoted the metastasis of breast cancer through sponging miR-148a-3p and miR-152-3p, which increases the expression of USF1 [37]. In another study, circIKBKB was seen to promote BC bone metastasis [38]. Additionally, fatty acid metabolism supports novel insights into BC patients' prognosis, suggesting that cell metabolism may trigger the progression of BC [39].

In this study, we determine whether circKIF4A can affect the growth and migration of breast cancer. It was found that circKIF4A was frequently upregulated in breast cancer [27]. Our results showed that circKIF4A was involved in the reprogramming of glucose metabolism in breast cancer. The absence of circKIF4A inhibited glucose uptake and lactate production in breast cancer cells, indicating that miR-335 may be blocked to inhibit breast carcinoma progression and liver metastasis by increasing the expression of glucose-metabolism-related proteins ALDOA and OCT4, which regulate the expression of HK2 and PKM2 protein. In clear cell renal cell carcinoma, miR-335 was shown to be downregulated and to be an important tumor suppressor [40]. In another study, miR-335 inhibition suppresses the bone metastases of small cell lung cancer via IGF-IR and RANKL pathways [41]. Hsa_circ_103973 promotes cervical cancer progression through miR-335 [42]. As a proven target of miR-335, ALDOA and OCT4 regulate glucose metabolism and homeostasis [25, 26, 43]. With the increasing incidence of drug-tolerant in various breast cancer subtypes [44–46], new therapies or diagnostics could be developed for distant metastasis based on the relationship between circKIF4A and glucose metabolism. Accordingly, our study found that circKIF4A is biologically active in BC and revealed the precise role of the circKIF4A-miR-335-ALDOA/OCT4-HK2/PKM2 axis in the metabolic reprogramming during the development of breast cancer and liver metastasis.

This study has some limitations. First, the relative expression of circKIF4A in BC, liver metastasis, and noncancer samples are from one single center with a small sample size, which may cause selection bias. Second, we need further experiments to verify the role of the circKIF4A-miR-335-ALDOA/OCT4-HK2/PKM2 axis in glucose metabolism.

## 5. Conclusions

Our study supported that circKIF4A plays an important role in BC tumorigenesis and liver metastasis via the circKIF4A-miR-335-ALDOA/OCT4-HK2/PKM2 axis, which could be intervened for BC treatment.

## Figures and Tables

**Figure 1:** circKIF4A is a circular RNA structure and its expression is elevated in breast cancer and liver metastasis. (a) circKIF4A expression in primary breast cancer and liver metastases compared to noncancer tissues. (b) The relative levels of circKIF4 expression in MCF-7, BT474, and HCC1806 cells. (c) RNase R assay was used to examine the circular structure of circKIF4. (d) The stability of circKIF4A was determined using actinomycin D treatment. Cell lines tested included MCF-7, BT474, and HCC1806. ^*∗*^*P* < 0.05; ^*∗∗*^*P* < 0.01; ^*∗∗∗∗*^*P* < 0.0001.

**Figure 2:** Silencing circKIF4A suppresses glucose metabolism and prevents breast cancer cells from metastasis. (a) Transfection with si-circKIF4A reduced glucose uptake. (b) A reduction in lactate production was observed when circKIF4A was silenced. (c) The ability of BC cells transfected with siRNAs to migrate and invade was measured using transwell migration (scale bar = 100 *μ*m), respectively. ^*∗*^*P* < 0.05; ^*∗∗*^*P* < 0.01.

**Figure 3:** circKIF4A acts as a sponge for miR-335. (a) The nucleocytoplasmic fraction assay revealed that circKIF4A is mainly localized in the cytoplasm, of BC cells. GAPDH was used as a cytoplasmic control and 18 S as a nuclear control. (b) Binding sites predicted for miR-335 in the circKIF4A sequence. (c) A dual luciferase reporter assay showed circKIF4A interacted with miR-335. (d) Based on RNA immunoprecipitation (RIP) assays, miR-335 was remarkably elevated in the MS2-circKIF4A-wt group. (e) Transfecting si-circKIF4A induced an increase in miR-335 expression. ^*∗∗*^*P* < 0.01.

**Figure 4:** circKIF4A regulates breast cancer metabolic reprogramming. (a) miR-335 expression in BC cell lines. (b) A comparison of miR-335 expression in primary BC and liver metastasis tissues as well as noncancer tissues. (c) The glucose uptake and lactate production amount were reduced after transfection with siRNA. (d) Identified miR-335-5p interacting sequences within the 3′-UTR of ALDOA and POU5F mRNAs. (e) The transfection of miR-335 mimics could remarkably suppress the mRNA expression of ALDOA/HK2 and OCT4/PKM2. (f) The introduction of miR-335 mimics decreases the protein expression of ALDOA/HK2 and OCT4/PKM2. ^*∗*^*P* < 0.05; ^*∗∗*^*P* < 0.01.

**Figure 5:** Cancer metastasis and tumor proliferation are promoted by CircKIF4A in vitro and in vivo. (a) Visible tumor nodules of liver metastasis. (b) Representative images of liver metastatic nodules. (c) Hematoxylin-eosin-stained sections of liver metastatic nodules (scale bar = 50 *μ*m). (d) Transfections with circKIF4A mimics increased glucose uptake and lactate production, which was reversed by the supplement of miR-335.

## Data Availability

The data used to support the findings of this study are available from the corresponding author upon request.

## References

[1] Sung H., Ferlay J., Siegel R. L. (2021). Global cancer statistics 2020: GLOBOCAN estimates of incidence and mortality worldwide for 36 cancers in 185 countries. *CA: A Cancer Journal for Clinicians*.

[2] Siegel R. L., Miller K. D., Fuchs H. E., Jemal A. (2021). Cancer statistics, 2021. *CA: A Cancer Journal for Clinicians*.

[3] He Z. Y., Wu S. G., Peng F. (2017). Up-regulation of RFC3 promotes triple negative breast cancer metastasis and is associated with poor prognosis via EMT. *Translational Oncology*.

[4] Adam R., Aloia T., Krissat J. (2006). Is liver resection justified for patients with hepatic metastases from breast cancer?. *Annals of Surgery*.

[5] Pockaj B. A., Wasif N., Dueck A. C. (2010). Metastasectomy and surgical resection of the primary tumor in patients with stage IV breast cancer: time for a second look?. *Annals of Surgical Oncology*.

[6] Zou Y., Hu X., Deng X. (2021). Distant lymph node metastases from breast cancer-is it time to review TNM cancer staging?. *JAMA Network Open*.

[7] Eng L. G., Dawood S., Sopik V. (2016). Ten-year survival in women with primary stage IV breast cancer. *Breast Cancer Research and Treatment*.

[8] Chen L. L., Yang L. (2015). Regulation of circRNA biogenesis. *RNA Biology*.

[9] Jeck W. R., Sorrentino J. A., Wang K. (2013). Circular RNAs are abundant, conserved, and associated with ALU repeats. *RNA*.

[10] Liu C. X., Chen L. L. (2022). Circular RNAs: characterization, cellular roles, and applications. *Cell*.

[11] Rong Z., Xu J., Shi S. (2021). Circular RNA in pancreatic cancer: a novel avenue for the roles of diagnosis and treatment. *Theranostics*.

[12] Xiao W., Zheng S., Zou Y. (2019). CircAHNAK1 inhibits proliferation and metastasis of triple-negative breast cancer by modulating miR-421 and RASA1. *Aging*.

[13] Li J., Sun D., Pu W., Wang J., Peng Y. (2020). Circular RNAs in cancer: biogenesis, function, and clinical significance. *Trends in Cancer*.

[14] Zou Y., Zheng S., Deng X. (2020). Diagnostic and prognostic value of circular RNA CDR1as/ciRS-7 for solid tumours: a systematic review and meta-analysis. *Journal of Cellular and Molecular Medicine*.

[15] Zou Y., Zheng S., Deng X. (2019). The role of circular RNA CDR1as/ciRS-7 in regulating tumor microenvironment: a pan-cancer analysis. *Biomolecules*.

[16] Lou J., Hao Y., Lin K. (2020). Circular RNA CDR1as disrupts the p53/MDM2 complex to inhibit Gliomagenesis. *Molecular Cancer*.

[17] Weng W., Wei Q., Toden S. (2017). Circular RNA ciRS-7-A promising prognostic biomarker and a potential therapeutic target in colorectal cancer. *Clinical Cancer Research*.

[18] Mao W., Wang K., Xu B. (2021). ciRS-7 is a prognostic biomarker and potential gene therapy target for renal cell carcinoma. *Molecular Cancer*.

[19] Yang Y., Gao X., Zhang M. (2018). Novel role of FBXW7 circular RNA in repressing glioma tumorigenesis. *Journal of the National Cancer Institute: Journal of the National Cancer Institute (1988)*.

[20] Ye F., Gao G., Zou Y. (2019). circFBXW7 inhibits malignant progression by sponging miR-197-3p and encoding a 185-aa protein in triple-negative breast cancer. *Molecular Therapy—Nucleic Acids*.

[21] Liu P., Zou Y., Li X. (2020). circGNB1 facilitates triple-negative breast cancer progression by regulating miR-141-5p-igf1r Axis. *Frontiers in Genetics*.

[22] Chen W., Zhang T., Bai Y. (2021). Upregulated circRAD18 promotes tumor progression by reprogramming glucose metabolism in papillary thyroid cancer. *Gland Surgery*.

[23] Zou Y., Zheng S., Xiao W. (2019). circRAD18 sponges miR-208a/3164 to promote triple-negative breast cancer progression through regulating IGF1 and FGF2 expression. *Carcinogenesis*.

[24] Tang H., Huang X., Wang J. (2019). circKIF4A acts as a prognostic factor and mediator to regulate the progression of triple-negative breast cancer. *Molecular Cancer*.

[25] Kuang Q., Liang Y., Zhuo Y. (2021). The ALDOA metabolism pathway as a potential target for regulation of prostate cancer proliferation. *OncoTargets and Therapy*.

[26] Marsboom G., Zhang G. F., Pohl-Avila N. (2016). Glutamine metabolism regulates the pluripotency transcription factor OCT4. *Cell Reports*.

[27] Shen Y., Xu J., Pan X. (2020). LncRNA KCNQ1OT1 sponges miR-34c-5p to promote osteosarcoma growth via ALDOA enhanced aerobic glycolysis. *Cell Death & Disease*.

[28] Cai S., Geng S., Jin F., Liu J., Qu C., Chen B. (2016). POU5F1/Oct-4 expression in breast cancer tissue is significantly associated with non-sentinel lymph node metastasis. *BMC Cancer*.

[29] Morfouace M., Lalier L., Oliver L. (2014). Control of glioma cell death and differentiation by PKM2-Oct4 interaction. *Cell Death & Disease*.

[30] Weiner H., Tompkins L., Keefer C. (2022). 70 Glycolytic substrates influence intracellular movement of PKM2 and OCT4 expression in bovine preimplantation embryos. *Reproduction, Fertility and Development*.

[31] Arnedos M., Vicier C., Loi S. (2015). Precision medicine for metastatic breast cancer--limitations and solutions. *Nature Reviews Clinical Oncology*.

[32] Kristensen L. S., Jakobsen T., Hager H., Kjems J. (2022). The emerging roles of circRNAs in cancer and oncology. *Nature Reviews Clinical Oncology*.

[33] Vo J. N., Cieslik M., Zhang Y. (2019). The landscape of circular RNA in cancer. *Cell*.

[34] Glažar P., Papavasileiou P., Rajewsky N. (2014). circBase: a database for circular RNAs. *RNA*.

[35] Zhang X. O., Dong R., Zhang Y. (2016). Diverse alternative back-splicing and alternative splicing landscape of circular RNAs. *Genome Research*.

[36] Kong Y., Yang L., Wei W. (2019). CircPLK1 sponges miR-296-5p to facilitate triple-negative breast cancer progression. *Epigenomics*.

[37] Zeng K., He B., Yang B. B. (2018). The pro-metastasis effect of circANKS1B in breast cancer. *Molecular Cancer*.

[38] Xu Y., Zhang S., Liao X. (2021). Circular RNA circIKBKB promotes breast cancer bone metastasis through sustaining NF-*κ*B/bone remodeling factors signaling. *Molecular Cancer*.

[39] Tang Y., Tian W., Xie J. (2022). Prognosis and dissection of immunosuppressive microenvironment in breast cancer based on fatty acid metabolism-related signature. *Frontiers in Immunology*.

[40] Zhang W., Liu R., Zhang L. (2022). Downregulation of miR-335 exhibited an oncogenic effect via promoting KDM3A/YAP1 networks in clear cell renal cell carcinoma. *Cancer Gene Therapy*.

[41] Gong M., Ma J., Guillemette R. (2014). miR-335 inhibits small cell lung cancer bone metastases via IGF-IR and RANKL pathways. *Molecular Cancer Research*.

[42] Zhu Y., Jiang X., Zhang S., Wang L., Zhou Q., Jiang J. (2020). Hsa_circ_103973 acts as a sponge of miR-335 to promote cervical cancer progression. *OncoTargets and Therapy*.

[43] Ji Y. Y., Song Y., Wang A. N. (2021). MiR-335-5p inhibits proliferation of Huh-7 liver cancer cells via targeting the Oct4/Akt pathway. *European Review for Medical and Pharmacological Sciences*.

[44] Zou Y., Zheng S., Xie X. (2022). N6-methyladenosine regulated FGFR4 attenuates ferroptotic cell death in recalcitrant HER2-positive breast cancer. *Nature Communications*.

[45] Chang C. A., Jen J., Jiang S. (2022). Ontogeny and vulnerabilities of drug-tolerant persisters in HER2^+^ breast cancer. *Cancer Discovery*.

[46] Slade D. (2020). PARP and PARG inhibitors in cancer treatment. *Genes & Development*.

